The article "Morpho-Physiological and Proteomic Analyses of Eucalyptus camaldulensis as a Bioremediator in Copper-Polluted Soil in Saudi Arabia" was retracted in 2020. Reasons: errors in the data; errors in the methods.

# Morpho-Physiological and Proteomic Analyses of *Eucalyptus camaldulensis* as a Bioremediator in Copper-Polluted Soil in Saudi Arabia

**DOI:** 10.3390/plants8020043

**Published:** 2019-02-15

**Authors:** Modhi O. Alotaibi, Afrah E. Mohammed, Taghreed A. Almutairi, Mudawi M. Elobeid

**Affiliations:** 1 Department of Biology, Faculty of Science, Princess Nourah bent Abdul-Rahman University, Riyadh 11474, Saudi Arabia; mouotaebe@pnu.edu.sa (M.O.A.); tag32-23@hotmail.com (T.A.A.); 2 Department of Silviculture, Faculty of Forestry, University of Khartoum, Khartoum North, Shambat 13314, Sudan; emudawi2828@hotmail.com

**Keywords:** *Eucalyptus camaldulensis*, copper, growth, proteomics, pollution

## Abstract

The present investigation aimed to assess the impact of copper (Cu) stress on the physiological and proteomic behavior of *Eucalyptus camaldulensis.* *E. camaldulensis* is likely a potential phytoremediator in areas vulnerable to Cu contamination, such as the industrial areas of Riyadh. To realize this objective, young seedlings of *E. camaldulensis* were potted in an open area with soil comprised of clay and sand. Different doses of Cu (30, 50, and 100 µM) were applied to the plants as CuSO_4_·5H_2_O for 6 weeks. Plant growth was monitored during the Cu exposure period, and morphological and physiological indicators were measured once a week to determine the growth rates. A proteomics study was also conducted to find out the influence of Cu stress on proteins. Our results showed that growth was negatively affected by Cu treatment, particularly at the highest concentrations. Moreover, using a proteomic analysis showed 26 targets involved in protein expression. Elevated levels of Cu increased the expression of 11 proteins and decreased the expression of 15 proteins. Changes were detected in proteins involved in photosynthesis, translation, transcription, metabolism, and antioxidant enzymes. Our findings provided insights into the molecular mechanisms related to Cu stress, in addition to its influence on the morphological and physiological attributes of *E. camaldulensis* seedlings. This investigation aimed to characterize the mechanism behind the impact of Cu stress on the plant.

## 1. Introduction

Today the globe is facing critical environmental crises, posing severe problems to humans and natural habitats [1]. Among such ecological complications is the stress in plants caused by water and soil contaminated with heavy metals, leading to stress in the overall food chain. Recently, a variety of factors have substantiated the pollution levels of air, water, and soil. Such factors include industrial activities, abandonment, sewage discarding practices, and the growth of cities, all posing toxic threats to living organisms [2,3]. Heavy metals are broadly recognized by their relatively high atomic masses (usually above 4 g/cm^3^), and are poisonous even at low concentrations [4,5]. For adequate plant development, some heavy metals are considered essential nutrients that play significant roles in plant life. However, accumulation of such metals in the environment has increased dramatically, often higher than that necessary for the plant’s growth. Under these elevated levels, all heavy metals have increased toxic effects and can be regarded as ecological impurities [6].

Many reports indicate plants are equipped with specialized tolerance mechanisms that mitigate the adverse effects of heavy metal exposure, although significant damage in plants, such as suppression of photosynthesis, was also observed as a consequence of elevated heavy metal exposure [7,8]. However, Maisto et al. [9] reported contrasting observations related to photosynthesis in *Quercus ilex* L. leaves when studying metal and polycyclic aromatic hydrocarbons (PAHs) as indicators of pollution.

The toxicity of heavy metals involves its binding to functional sites in biologically vital molecules (enzymes), disturbing cell integrity by changing proteins and nucleic acids, as well as disrupting other important metabolites in the cell [10]. Among the heavy metals, copper (Cu^2+^) is a toxic metal. In the current investigation we focus on Cu^2+^. Cu^2+^ is a redox-active transition ion and a necessary micro-element for plant development [11], however, it can be considered a toxic element when its concentrations in plant tissue exceeds that of the optimum requirement [12,13,14]. The positive influence of Cu on plant growth has long been observed, and has been well-recognized when fungicides containing Cu salts are used [15]. However, the common and continued use of fungicides in cultivated areas has led to a high accumulation of Cu, putting both the ecological value and the fertility of the soil at hazardous levels [16]. Plants exposed to heavy metals may also be subjected to a widespread range of physiological and biochemical alterations [17].

Auto-oxidation and the Fenton reaction usually lead to development of reactive oxygen species (ROS), leading to the block of important biomolecules. Movement of metal ions from such biomolecules is the main mechanism of heavy metal accumulation in plant tissues [2]. Furthermore, in our post-genomic era, proteomics is a well-known technique to study protein expression in an organism through its genome [18,19]. Moreover, plant stress responses, and adaptation to the stress caused by heavy metals, are frequently associated with alterations in the proteome [17]. Proteomics can be used as a powerful technique to uncover differences in cell, tissue, organ, and organelle protein levels, including the profiles under several heavy metal stress environments [20]. The literature also mentions that proteomics help in detecting the target proteins involved in heavy metal detoxification. Recent studies confirmed the increments of defense protein involved in ROS scavenging and in maintaining redox homeostasis in heavy metal stressed plants [21,22]. In an early study by Bona et al. [23], the response of *Cannabis sativa* roots to Cu stress was reported. Their findings revealed variations in the protein expression pattern for reinstating cellular homeostasis, where two proteins were suppressed, seven proteins were down regulated, and five proteins were up regulated. Some proteomic studies were focused on Cu stress in *Arabidopsis thaliana* [24], *Cannabis sativa* roots L. [23], *Oryza sativa* [25], and *Agrostis capillaris* [26].

Plants react differentially to heavy metal stresses according to their species, the metal type, and metal concentration [27]. Therefore, the molecular mechanisms of plant responses are needed using proteomic studies under Cu stress. In the current study we have tried to uncover the relationship between Cu stress and the molecular response in *E. camaldulensis* seedlings. *E. camaldulensis* has been used in the current study because it is abundant in Riyadh industrial areas. These industries might be the main reason for environmental contamination, especially in industries where production of fertilizer involves Cu and leads to its bioavailability and abundance in the environment. Furthermore, *E. camaldulensis* is characterized by its fast growth rate, relatively large biomass, extensive root system, and its tolerance to a wide spectrum of soil conditions [28]. Therefore, the present investigation was based on the assumption that *E. camaldulensis* would fit as a good candidate plant species for environmental clean-up in sites contaminated with heavy metals. This hypothesis might be well supported by Assareh et al. [29]. Nevertheless, its molecular response to Cu stress is still vague. Proteomics results and physiological responses from the current study might improve our understanding of *E. camaldulensis* and its response to Cu stress. A thorough understanding of the plant’s stress response to heavy metals could support the identification of tolerance proteins or genes, and the development of a detoxification tool [30].

## 2. Materials and Methods

### 2.1. Ethics Statement

Determination of the target species chosen for this study was performed by collecting materials of several plant species from three different locations (Riyadh industrial area, landfill near Nazeem, and Thumamah) in Riyadh (N 38.24°, E 43.46°), Saudi Arabia. No collection specifications were obligatory for these locations. Plants used in the current study are public and non-protected types. The candidate plant species chosen for the current investigation is *E. Camaldulensis* due to its availability in the three different locations.

### 2.2. Material Collection and Treatment

*E. camaldulensis* seedlings (three months old) were provided from a commercial nursery in Riyadh, May 2017. Similar genetic backgrounds were expected since plants were collected from the same source. The seedlings were acclimated to a greenhouse (temperature 28–35 °C, photoperiod 12 hours per day). *E. camaldulensis* seedlings were placed into pots (16 cm diameter) containing a soil mixture of clay:sand in a 1:2 ratio. The experimental plants were exposed to a wide range of Cu concentrations (100, 50, and 30 µM of Cu, applied as CuSO_4_·5H_2_O for a period of six weeks). Each Cu treatment was comprised of four replicates. Shoots and roots per plant were cut, washed in deionized water, placed in airtight plastic bags, and then kept at −80 °C for additional study.

### 2.3. Growth and Physiological Performance

During the experimental period, growth indicators were monitored weekly (height, stem collar width, and leaf formation), and the relative growth rates were calculated. The relative water content of the leaves, and fresh weights of both shoot and root were determined gravimetrically following termination of the experiment. Plant samples were oven-dried for one week at 60 °C to achieve a constant weight for determining shoot and root dry mass.

### 2.4. Determination of Relative Water Content

For determination of relative water content in the plant under Cu stress, leaf tissues were taken to determine the relative water content, according to Morgan [31], with the aid of the following equation:

$$\mathrm{RWC}\left(\%\right)=\frac{\left(\mathrm{fresh}\;\mathrm{weight}\;-\;\mathrm{dry}\;\mathrm{weight}\right)}{\left(\mathrm{sturated}\;\mathrm{weight}\;-\;\mathrm{dry}\;\mathrm{weight}\right)}\times 100$$

### 2.5. Determination of Chlorophyll Content

Leaf samples were collected and frozen immediately. Chlorophyll content was determined when 5 mL of 80% acetone was added to a 0.5 g leaf sample and measured using spectrophotometer. Resulting data were calculated as mg/g Fresh weight [32]. Chlorophyll content data was presented as mean ± SD for three replicates.

### 2.6. Determination of Copper (Cu) Concentration

Cu concentrations in leaves and root tissues were determined using atomic absorption spectroscopy (NOVA 300, Analytik, Jena, Germany) according to Fu et al. [33]. Dry plant samples were milled to a fine powder, then digested using perchloric acid and nitric acid in a ratio of 13:87 by volume. Thereafter, 5% of HNO_3_ was used to dissolve the digest for Cu quantification.

### 2.7. Protein Extraction from Plant Leaves

For the determination of protein, liquid nitrogen was used for milling the frozen leaves using a mortar and pestle. The protein extraction procedure was done according to Roy et al. [34]. To perform two-dimensional gel electrophoresis (2-DE), a trichloroacetic acid (TCA)/acetone protocol was used. Two technical replicates per sample were prepared.

### 2.8. Trichloroacetic Acid (TCA)/Acetone Protocol

Leaf powders from the control plants (3 g) and the Cu-treated plants (100 µM) were placed in 10 mL of ice-cold 10% TCA in 0.07% (*v*/*v*) acetone and 2-mercaptoethanol (2-ME). The homogenate was sonicated for 10 min and incubated for 1 h at −20 °C. The pellet was separated after centrifugation at 4 °C for 20 min, washed with ice-cold acetone (0.07% (*v*/*v*) 2-ME) twice, and then centrifuged at 4 °C and dehydrated. Thereafter, dried samples were lysed using buffer (8 M urea, 2 M thiourea, 5% CHAPS, and 2 mM tributylphosphine), incubated for 60 min at 25 °C, and centrifuged at 20,000 rpm for 20 min. Thereafter, protein concentration was determined using the Bradford (Bio-Rad) method [35].

### 2.9. Two-Dimensional Gel Electrophoresis (2-DE) Protein Gel Electrophoresis

A gel electrophoresis technique (two-dimensional isoelectric focusing) was performed utilizing a Bio-Rad PROTEAN IEF (isoelectric focusing) cell on an IPG strip with a length of 24 cm and pH 5–8 (Bio-Rad, Richmond, CA, USA). For protein dilution, 300 lg total protein was diluted with a rehydration solution (8 M urea, 4% CHAPS, 1% DTT, 0.2% IPG buffer (pH 5–8), and 0.001% bromophenol blue) to 420 ll. Active rehydration was done by loading the samples into the IEF tray at 20 °C for 13 h, followed by 250 V for 60 min. Subsequently, a linear increase of voltage was applied to 10,000 V for a period of four hours, with isoelectric focusing operated at 20 °C for 90,000 VH. Following IEF separation, strips were equilibrated for 15 min in an equilibration buffer (6 M urea, 0.375 M Tris–HCl (pH 8.8), 20% glycerol, 2% SDS, and 2% DTT), then re-equilibrated for 15 min using the same buffer, except that DTT was replaced by 2.5% iodoacetamide. The 2-D SDS electrophoresis was done on 12.5% (*w*/*v*) horizontal slab gels using a Bio-Rad PROTEAN PLUS horizontal Dodeca cell at a temperature of 18 °C. For application of SDS–PAGE, voltage was fixed at 100 V for 60 min, then increased to 200 V until the bromophenol blue frontier was detected at the gel bottom.

### 2.10. Protein Imaging

For the purpose of staining protein spots, an image scanner (HP Scanjet G 4010) was used and the analysis was performed using the Progenesis Same Spot software version 3.0 (Nonlinear Dynamics Ltd.). Two replicates from both control and Cu-treated gels were used to carry out the match set with the selected master gels. Student’s t-test (*p* ≤ 0.05) was used to find out differences in the abundance between spots. For MS (mass spectrometry) identification, protein spots with > 2-fold changes were used.

### 2.11. Bioinformatics Analysis of the Identified Proteins

Proteins identified in the current investigation were clustered according to Colak et al. [36] using DAVID gene ontology (GO) enrichment analysis bioinformatics tools. Fold changes of identified proteins at Cu treatment (100 µM) compared to control are presented.

### 2.12. Statistical Analysis

The current data was statistically processed using JMP statistical program (SAS Institute, Inc., Cary, North Carolina, USA). Trials were set using four plants per Cu treatment. A one-way ANOVA was used, and means were separated by a Tukey-test at *p* ≤ 0.05 significance, which is denoted by dissimilar letters. Figures were prepared using Origin software.

## 3. Results and Discussion

### 3.1. Changes in Plant Morphology

With progressive increases of Cu treatment, leaf chlorosis was noticeable after five weeks from the commencement of Cu treatment in the *E. camaldulensis* seedlings. The degree of chlorosis was more intense in plants that received 100 µM compared to those treated with low Cu concentrations (30 and 50 µM). In addition, the leaves on the plant that received the highest Cu dose started to droop and saw increasing discoloration. Early studies indicated that phytotoxicity induced by excessive Cu uptake may lead to plant growth suppression, membrane lipid peroxidation, leaf chlorosis, and necrosis [24,37]. Some of these results and observations are in agreement with our current findings.

### 3.2. Influence of Cu on Plant Growth

Exposure of *E. camaldulensis* to Cu caused no effect on shoot height both at 30 and 50 µM concentrations; however, seedlings that received the highest dose (100 µM) exhibited significant reductions in their shoot height growth rates compared to untreated controls (Figure 1a). A similar response pattern was also observed in both stem diameter (Figure 1b) and leaf formation (Figure 1c). Furthermore, data showed higher Cu concentrations in roots relative to that in the shoots (Figure 1d).

The observed reduction in plant growth might be attributed to the inhibitory impact of the metal on the metabolic processes responsible for growth and development, which is in agreement with many other previous studies [9,14,38]. Furthermore, quantitative analysis showed that relative water content, chlorophyll content, shoot and root fresh weight, and shoot and root dry weight of seedlings treated with the highest dose (100 µM) were significantly reduced by 33.3%, 54.8%, 36.5%, 42.5%, 40.7%, and 33.3% respectively, relative to those of the control (Table 1). On the other hand, similar trends in observations and reductions were noticed for shoot and root fresh weight and shoot and root dry weight for *O. glazioviana* in response to Cu stress [27]. The perturbation in the biomass production in both shoot and root might be linked to the effect of Cu on cell division, which retarded normal cell growth and development [39]. The diminishing effect of Cu on chlorophyll content and remarkable reduction in relative leaf water content might be a consequence of Cu stress, as reported in other studies [40,41,42]. Mostofa et al. [41] stated that Cu stress induced a reduction in rice seedling growth, which might be due to the disruptive interference Cu has in protein and plant metabolism. Addition of Cu to *E. camaldulensis* seedlings was found to increase the Cu level in the plant tissues, with the root retaining more Cu relative to the shoot (Figure 1d), which indicates that roots are the main site for the accumulation of Cu. This observation conformed with several former reports in rice and beans [41,43].

Different studies have indicated that Cu is a detrimental metal that interferes with a plant’s morphological, physiological, and proteomic characteristics because Cu is highly toxic to the plant [44,45,46]. Fold changes in protein and protein expression in relation to Cu stress are introduced in Table 2. Twenty six (26) proteins were identified under Cu stress from the leaves of *E. camaldulensis*—11 saw increased protein expression and 15 saw decreased protein expression.

### 3.3. Classification of Identified Proteins

The 26 differentially expressed proteins were identified and the UniProt database was used. Figure 2 illustrates the protein gel images, and Figure 3 shows the abundance patterns of different separated proteins. Figure 4 shows the functional classes of the identified proteins with respect to their biological functions (Figure 4a,b) and cellular constituents (Figure 4c).

### 3.4. Changes in Proteomic Profile

The current investigation was designed to explore the possible mechanisms for the alterations seen in the plant protein when affected by Cu. The leaf proteome was tested using 2D-GE. Soluble proteins were determined from leaf tissues of both the treated and control plants. The experiment was replicated twice and identified 200 protein spots. Image analyses quantified 26 proteins expressing greater than a 1.5-fold increase in concentration. Out of the 26 differentially expressed proteins, 11 proteins increased expression, whereas the remaining 15 proteins assumed a decrease in the treated sample relative to controls. Figure 3 represents the separated proteins as a comparison between control and treated plants.

The separated proteins for the plants pre-treated with Cu were categorized in different groups according to molecular functions, including metabolic processes (45.8%), photosynthesis (16.7%), anti-oxidant enzymes (8.3%), transcription and translation processes (25%), and other unknown functions (15.5%). Cu stress may affect protein metabolism, which leads to a reduction in the protein concentration [47]. Different biological functions for such separated proteins might point to the complex plant processes observed under Cu stress conditions.

#### 3.4.1. Photosynthetic Proteins

It is well known that photosynthesis is the most important biological process in plants, and this process is extremely sensitive to various stress conditions. A high accumulation of heavy metals inhibits the plant’s growth and development, in addition to its effect on the photosynthetic products [39]. Previous investigations have shown that elevated levels of Cu stress adversely influence the physiological and biochemical processes, such as photosynthesis, metabolism of nitrogen, and element uptake in plants [13,48]. In the current study, several photosynthesis-related proteins were significantly reduced in Cu-stressed plants, such as rubisco (large and small sub-units). Photosynthesis-related proteins were also decreased by Cd stress in *Brassica juncea* [49,50], and had a damaging effect on vital activities, including photosynthesis, in *Zea mays* [51]. However, a recent investigation provided sufficient evidence, where photosynthetic responses to Cd and Pb stress in cardoon plant varieties were studied, to indicate that the effect of heavy metals on plants is species-specific [52].

Our findings also revealed that photosystem II was down-regulated. Similar response patterns have also been reported for other metals, such as Cd stress in sorghum [34]. The light-dependent photosynthesis reaction cytochrome b6 was negatively impacted by Cu stress. Similar observations were also noted by Hego et al. [26] when they studied the leaves of Cu-sensitive and Cu-tolerant *Agrostis cappilaris*. Alterations in photosynthetic electron transport chain components in response to stress may occur in the proteins involved cytochrome b6f [53]. Therefore, light-dependent (cytochrome b) and independent (rubisco) photosynthetic reactions were decreased, or negatively affected, by excess Cu in the leaves of *Eucalyptus camaldulensis.* This indicates damage in the photosynthesis mechanism since rubisco is the key enzyme responsible for CO_2_ assimilation during the dark reaction phase.

#### 3.4.2. Antioxidant Enzymes and Related Proteins

Plant exposure to Cu may generate ROS, leading to oxidative stress and cell mortality [54]. Plants may develop defense mechanisms to mitigate and alleviate such effects, and prevent cell oxidation [55]. These mechanisms might be associated with enzymatic compounds, such as peroxidases and superoxide dismutase, that play an important ROS scavenging role. Some studies have shown that metal stress (such as Cd) may impair the antioxidant system in plants; therefore, ROS will be induced and will directly react with cellular components and organelles [56]. The anticipated accumulation of ROS during Cu stress may lead to the generation of high levels of antioxidant enzymes. Our study revealed that enzymes related to peroxidase detoxification were down regulated, however the Cu/Zn superoxide dismutase showed increased accumulation during Cu treatment. A comparable pattern for SOD activity was also noted by Li et al. [46] when they studied *Eichhornia crassipes* and *Pistatia stratiotes* under Cd stress. Peroxidase down-regulation, observed for the Cu-stressed plants in the current study, might lead to speculation that the peroxidase was consumed during the defense process. Although, in a recent study [27], peroxidase accumulation in the roots of *Oenthera glazioviana* under Cu stress was shown.

In conclusion, alteration in the expression of ROS detoxification-related enzymes was apparent in the current study for peroxidase and Cu/Zn-SOD, highlighting the functions they display in cell protection.

#### 3.4.3. Glycolysis and Carbohydrate Metabolism Related Proteins

The current investigation identified six proteins: Glyceraldehyde-3-phosphate dehydrogenase, Fructose-bisphosphate aldolase, Sucrose synthase, Phosphoribulokinase, Starch synthase_ chloroplastic/amyloplastic, and Phospholipase D. Glycolytic glyceraldehyde-3-phosphate (GADPH) dehydrogenase is the major redox controller in metabolic process [57]. In energy metabolism the CA cycle is a key pathway for ATP synthesis, and responds to stressed environments through respiratory oxidation [58]. The current findings showed up-regulation of GADPH in plants exposed to Cu, as it could be involved in the response to biotic stress in the plant by glycolysis [59]. Similar increments of GADPH in *A. thaliana* under Cd stress was observed [60]. On the other hand, reduction of GADPH was reported when barley and rice were subjected to stress conditions with salt [61], and Poplar root when treated with Cd [62]. Furthermore, fructose-bisphosphate aldolase, a catalyst involved in splitting fructose-1-6-bisphosphate into D-glyceraldehyde-3-phosphate [63], is involved in glycolysis in the cytoplasm and in the Calvin cycle. Fructose-bisphosphate aldolase decreased in the current study in response to Cu stress, as well as in *Ectocarpus siliculosus* isolated from Cu-contaminated soil [64]. Down-regulation of malate dehydrogenase (MDH) in the current study was supported by Kamal et al., [65] when he studied salt stress in wheat. The significance of MDH in Brachypodium seedling roots was reported as an adaptation response to a biotic stress by Chen et al. [66]. The down-regulation of MDH was observed during the first 3 days, but at 4 days it responded to Cd and osmotic stresses. Malte dehydrogenase may enhance a plant’s resistance to salt and Al stress since it increases the malic acid levels [67].

#### 3.4.4. Energy and Carbohydrate Metabolism Proteins

The beta subunit of ATP synthase identified in the current investigation was down-regulated. It is an integrated protein associated with ATP hydrolysis and proton movement, providing electrochemical compounds [68]. Therefore, an increased production of ATP in response to Cu stress was expected. In a recent work, stimulation of ATPases in *Agrostis capillaris* leaves under Cu stress was noted [26], whereas other studies using tomato and wheat plants showed that ATPases were reduced in response to salt stress [69].

#### 3.4.5. Proteins Involved in Transcription and Translation

Suppression of proteins and enzyme inactivation induced by heavy metal stress may affect cellular homeostasis [50]. Damaging effects on many cellular processes might be a consequence of the limitations in different gene regulators due to heavy metal stress [70]. In the present investigation, translational proteins such as 30S ribosomal S14, 30S ribosomal S15, eukaryotic translation initiation factor 5A (eIF5A), and RNA-dependent RNA polymerase were down-regulated in *E. camaldulensis* leaves under 100 µM Cu treatment; however, elongation factor Tu was up-regulated. The eIF5A protein is a eukaryotic protein that contains hypusine amino acid; it has an important role as the translation initiation factor in RNA metabolism [71], and translation elongation [72]. Increased expression of eIF5A in plants related to abiotic stress was noted [73]. Currently, down regulation of eIF5A was noted (Table 2). Results were in line with Chen et al. [45] when he studied the behavior of two rice (*Oryza sativa* L.) cultivar roots under Cu stress. The main subunit of ribosomes in mitochondria and chloroplasts is 30S [74]. This protein is involved in the translation process. 30S ribosomal protein S14 and S15 in chloroplasts were down-regulated in the current study under 100 µM Cu treatment in *E. camaldulensis* leaves. The same observations were also detected for Poplar leaves under Cd stress [75]. Genes related to translation and transcription can be expressed and regulated when the plant is subjected to adverse environmental conditions, leading to adaptation [76]. In the higher plants, the translational elongation step is mainly regulated by elongation factors. Down-regulation of the putative elongation factor 2 in rice under Cu stress conditions was noted [45], however, the current study detected up-regulation of elongation factors for *E. camaldulensis* leaves under Cu stress. RNA-dependent RNA polymerases (RdRp) are enzymes that amplify microRNAs in eukaryotes [77], and protect plants against pathogenic agents [78]. In the current study, down regulation of RdRp was observed. Heat stress showed a decrease in mutant *rdr2* for the gene encoding RdRp2 and *dcl3* in Arabidopsis [79].

## 4. Conclusions

As stated previously, accumulation of heavy metals in plants may lead to a variety of deleterious effects in growth and development via perturbations in metabolic network. Cu can be highly toxic to plants when taken in excessive amounts. Hence, the present investigation was undertaken to highlight the alterations in plant metabolism that take place in *E. camaldulensis* as it responds to Cu stress exposure. Several stress indicators, together with proteomic studies, were analyzed under Cu stress to diagnose the effects. The damaging effects of Cu on growth and biomass elements for the *E. camaldulensis* seedlings was apparent, with the response being most pronounced under the elevated Cu level of 100 µM. Proteomic analysis performed in this investigation identified 26 proteins related to various metabolic functions, and such proteins were expressed at different availability levels under Cu stress conditions. The majority of the characterized proteins were mainly stress proteins as well as metabolism and regulatory proteins. Results obtained from the proteomic analysis has provided significant clues on how *E. camaldulensis* responds to Cu stress to achieve homeostasis.

Our findings showed a significant influence of Cu on protein metabolism, as attested by the inhibition of protein function. Proteomic analysis revealed the presence of special stress-related proteins, which can be speculated to assist *E. camaldulensis* seedlings in handling exposure to Cu exposure. In the future, it would be beneficial to further investigate the long-term effects of Cu on *E. camaldulensis*. Results of long-term investigations would enhance our understanding of the responsiveness of *E. camaldulensis* under various Cu toxicity levels.

## Figures and Tables

**Figure 1:** Effects of Cu stress on (**A**) shoot height, (**B**) stem diameter, (**C**) leaf formation, and (**D**) Cu concentration in the leaves and roots of *E. camaldulensis* seedlings. Different letters indicate significant differences at *p* < 0.05. Each experiment was performed in four replicates.

**Figure 2:** Representative images gel spots, indicating protein changes among (**A**) control plants and (**B**) treated plants. Separated proteins are highlighted in Table 2.

**Figure 3:** Principal component analysis of 26 differentially expressed proteins. (ANOVA *P* < 0.05, and > 2-fold change). (**A**) control and (**B**) treated.

**Figure 4:** Functional classification of identified proteins from leaves of *E. camaldulensis*. Proteins were categorized based on the information from iProClass databases and gene ontology. **A** and **B** are biological processes, and **C** is the cellular components.

**Table 1:** Effect of copper (Cu) stress on growth characteristics of *E. camaldulensis*. Statistically significant differences are indicated with stars: (*) *p* < 0.05 or (**) *p* < 0.01. Data are given as means ± standard deviation (SD).

Physiological Index	Control	Cu (30 µM)	Cu (50 µM)	Cu (100 µM)	Change Fold (Control/Cu 100 µM)
Relative water content (%)	84 ± 2.5	73 ± 3.1	70 ± 2.9	56 ± 2.6 *	1.5
Chlorophyll content (mg/g)	3.1 ± 0.12	2.5 ± 0.3	2.1 ± 0.1	1.4 ± 0.1 *	2.21
Shoot fresh weight (g·plant−1)	2.00 ± 0.01	1.98 ± 0.1	1.65 ± 0.01	1.27 ± 0.09 *	1.57
Root fresh weight (g·plant−1)	1.01 ± 0.01	0.92 ± 0.01	0.72 ± 0.02	0.58 ± 0.01 *	1.74
Shoot dry weight (g·plant−1)	0.27 ± 0.01	0.23 ± 0.02	0.19 ± 0.01	0.16 ± 0.01 *	1.68
Root dry weight (g·plant−1)	0.03 ± 0.002	0.03 ± 0.001	0.02 ± 0.001	0.02 ± 0.001 **	1.5

**Table 2:** List of principal component analysis of differentially expressed proteins by Cu stress in the leaves of *E. camaldulensis*, using MALDI-TOF-TOF mass spectrometry.

Accession	Description	Gene	Control	Treated
**Photosynthesis**				
tr|A7U3N0|A7U3N0_EUCGL	Ribulose bisphosphate carboxylase large chain (Fragment)	GN=rbcL PE=3 SV=1	7379.896	1713.233
tr|D1MZ07|D1MZ07_EUCGL; tr|A0A059A414|A0A059A414_EUCGR; tr|A0A059AHP3|A0A059AHP3_EUCGR; tr|A0A059AI83|A0A059AI83_EUCGR; tr|A0A059AIQ7|A0A059AIQ7_EU	Ribulose bisphosphate carboxylase small chain	GN=EgRBCS2 PE=2 SV=1	13005.96	6464.88
tr|A0A2N9QPM6|A0A2N9QPM6_9ROSA; tr|T1QP85|T1QP85	Photosystem II D2 protein	GN=psbD PE=3 SV=1	31698.33	14556.42
sp|Q49KW8|CYB6_EUCGG	Cytochrome b6	GN=petB PE=3 SV=1	1029.958	550.3955
**Translation and transcription**				
tr|A0A2N9QPN7|A0A2N9QPN7_9ROSA	30S ribosomal protein S14_ chloroplastic	GN=rps14 PE=3 SV=1	827.5739	286.2062
tr|A0A2K8GMY3|A0A2K8GMY3_9ROSA	30S ribosomal protein S15_ chloroplastic	GN=rps15 PE=3 SV=1	366.9244	154.6282
tr|A0A059AZP2|A0A059AZP2_EUCGR	Elongation factor Tu	GN=EUGRSUZ_H01524 PE=3 SV=1	433.0593	911.957
tr|A0A059CKD9|A0A059CKD9_EUCGR	Eukaryotic translation initiation factor 5A	GN=EUGRSUZ_C00350 PE=3 SV=1	2096.565	1001.485
tr|A0A059BE60|A0A059BE60_EUCGR	RNA-dependent RNA polymerase	GN=EUGRSUZ_G02093 PE=3 SV=1	2019.472	826.6111
tr|A0A1S6XZH0|A0A1S6XZH0_EUCGL	C-repeat binding factor	GN=CBF1d PE=2 SV=1	2137.21	7867.328
**Antioxidant enzyme**				
tr|A0A059B660|A0A059B660_EUCGR; tr|A0A059B6P5|A0A059B6P5_EUCGR; tr|A0A059B713|A0A059B713_EUCGR	Superoxide dismutase [Cu-Zn]	GN=EUGRSUZ_H04426 PE=3 SV=1	3380.004	9448.107
tr|A0A059CT24|A0A059CT24_EUCGR	Peroxidase	GN=EUGRSUZ_C02744 PE=3 SV=1	1737.219	751.3391
**Metabolism process** **Energy and carbohydrate metabolism**				
sp|Q49KZ1|ATPB_EUCGG	ATP synthase subunit beta_ chloroplastic	GN=atpB PE=3 SV=1	51102.71	33223.95
tr|A0A2K8GMV7|A0A2K8GMV7_9ROSA	ATP synthase subunit	GN=atpB PE=3 SV=1	23006.91	
sp|Q49KZ2|ATPE_EUCGG	ATP synthase epsilon chain_ chloroplastic	GN=atpE PE=3 SV=1	7304.724	4168.356
**Glycolysis and carbohydrate metabolism**				
tr|A0A059B8M0|A0A059B8M0_EUCGR	Glyceraldehyde-3-phosphate dehydrogenase (Fragment)	GN=EUGRSUZ_H04673 PE=3 SV=1	1885.399	5275.84
tr|A0A059A4U5|A0A059A4U5_EUCGR; tr|A0A059A3P2|A0A059A3P2_EUCGR	Fructose-bisphosphate aldolase	GN=EUGRSUZ_K02073 PE=3 SV=1	2140.208	4374.579
tr|A0A059C2Y2|A0A059C2Y2_EUCGR; tr|A0A059C3I0|A0A059C3I0_EUCGR	Phosphoribulokinase	GN=EUGRSUZ_E01261 PE=3 SV=1	62215.04	30478.44
tr|I0IK58|I0IK58_9MYRT; tr|I0IK59|I0IK59_9MYRT	Sucrose synthase (Fragment)	GN=SuSy1 PE=3 SV=1	632.5789	1286.607
tr|A0A059C344|A0A059C344_EUCGR	Starch synthase_ chloroplastic/amyloplastic	GN=EUGRSUZ_E01068 PE=3 SV=1	1051.751	294.2494
tr|A0A059BWS2|A0A059BWS2_EUCGR; tr|A0A059BX43|A0A059BX43_EUCGR	Phospholipase D	GN=EUGRSUZ_F03862 PE=3 SV=1	439.2654	200.1259
tr|A0A059BV12|A0A059BV12_EUCGR	Malate dehydrogenase	GN=EUGRSUZ_F03251 PE=3 SV=1	947.0006	2298.791
sp|P46487|MDHM_EUCGU	Malate dehydrogenase_ mitochondrial	GN=MDH PE=2 SV=1	6368.574	2733.391
**Unknown**				
tr|A0A059DFL1|A0A059DFL1_EUCGR	Purple acid phosphatase	GN=EUGRSUZ_A01512 PE=3 SV=1	7115.349	15029.53
tr|A0A059BJT7|A0A059BJT7_EUCGR	Patatin	GN=EUGRSUZ_F00259 PE=3 SV=1	14.78243	618.4795
tr|A0A059BV73|A0A059BV73_EUCGR	Probable bifunctional methylthioribulose-1-phosphate dehydratase/enolase-phosphatase E1	GN=EUGRSUZ_F03307 PE=3 SV=1	2655.225	777.6948
